RETRACTED

# EDTA Combined with C-Pilot Files and Microultrasound for Root Canal Calcification: Dredging Effect and Safety Analysis

**DOI:** 10.1155/2022/1911448

**Published:** 2022-10-11

**Authors:** Ting Chu, Xiufeng Ni, Yanhua Zhu

**Affiliations:** ^1^Department of Stomatology, Zhenjiang First People's Hospital Affiliated to Jiangsu University, Zhenjiang, Jiangsu 212002, China; ^2^Department of Stomatology, Xiaoshan Traditional Chinese Medical Hospital, Hangzhou, Zhejiang 311200, China

## Abstract

**Objective:**

This paper discussed the dredging effect and safety of ethylenediaminetetraacetic acid (EDTA) combined with C-pilot files and microultrasound (mUS) on root canal calcification.

**Methods:**

From October 2021 to January 2022, 132 patients with calcified root canals treated in our hospital were selected as the research subjects. Among them, 64 cases who received EDTA combined with C-pilot Files and mUS plus ultrasonic instruments to dredge calcified root canals were regarded as the research group (RG), and another 68 cases given ultrasonic instruments plus C-pilot files were regarded as the control group (CG). The root canal dredging time was recorded, and the dredging success rate and total success rate of different tooth positions and calcification sites were compared between groups. The clinical efficacy was assessed 6 months after treatment. Pain severity was evaluated by the Pain Intensity Numerical Rating Scale (PI-NRS) before (*T*0), during (*T*1), and after treatment (*T*2). Finally, the incidence of adverse reactions within one week after treatment was counted.

**Results:**

RG was observed with statistically higher success rates of root canal dredging in different tooth positions and calcified sites than CG (*P* < 0.05). Besides, the total effective rate of treatment was 92.19% in RG, which was also higher compared with CG, while the root canal dredging time in RG was shorter than that in CG (*P* < 0.05). Increased NRS scores were found in both groups at *T*1, and the score in RG was significantly lower compared with that in CG. At *T*2, both groups showed a lower PI-NRS score than *T*1 but higher than *T*0, and the score at *T*2 was also lower in RG as compared to CG (*P* < 0.05). Moreover, the reduced incidence of adverse reactions were observed in RG compared with CG (*P* < 0.05).

**Conclusions:**

EDTA combined with C-pilot files and mUS can effectively improve the dredging success rate of root canals obstructed by calcification, shorten the dredging time, and improve patient comfort, which is an effective method for clinical dredging of calcification obstructed root canals.

## 1. Introduction

Root canal therapy is currently the most effective means to treat pulpal and periapical diseases. However, as people grow older, the root canal will undergo physiological changes, the pulp cavity, and root canal will change, and the secondary dentin will be formed continuously, leading to the gradual tapering and even atresia of the root canal; meanwhile, the filled teeth will stimulate the dental pulp, which causes the formation of restorative dentin that will also stimulate the dental pulp to form root canal calcification [1, 2]. Unclogging the root canal is the key to achieving an effective root canal treatment [3]. However, for root canal calcification, the traditional treatment is not only time consuming and laborious but also induces obvious pain, resulting in low cooperation degree and a high rate of treatment failure [4]. There are emerging clinical treatments for root canal calcification as medical technology advances, and it is of great significance to find out the effective treatment means among them to improve root canal therapy [5].

RETRACTED

Ethylenediaminetetraacetic acid (EDTA) combined with C-pilot files and microultrasound (mUS) has been widely used in the clinical treatment of root canal calcification in recent years [6]. Studies have shown that EDTA has a good dissolving effect on calcified substances, and the C-pilot file is harder and easier to enter into small gaps, thus achieving the purpose of dredging root canals [7]. At the same time, the continuous progress of minimally invasive technology has enabled the gradual application of root canal microultrasonic technology to dental treatment. Under the magnification of the microscope, the cutting and oscillation performed with the help of ultrasonic instruments can effectively remove calcified substances in root canals [8]. The purpose of this study was to explore the dredging effect and safety of EDTA combined with C-pilot files and mUS on root canal calcification, so as to provide reliable and effective clinical theoretical guidance for future clinical treatment.

## 2. Materials and Methods

### 2.1. Study Area

The study was conducted from October 2021 to July 2022.

### 2.2. Data Acquisition

This research selected 132 cases of calcified dental root canals treated between October 2021 and January 2022, including 82 males and 50 females. Among which, 64 cases with the mean age of 46.34 ± 4.62 (research group (RG)) receiving EDTA combined with C-pilot Files and mUS plus ultrasonic instruments for calcified root canal dredging, and another 68 cases with the mean age of 47.28 ± 4.53 (control group (CG)) treated with ultrasonic instruments combined with C-pilot files. This study was approved by the Ethics Committee of our hospital and conducted in strict compliance with the Declaration of Helsinki, and all subjects signed the informed consent.

RETRACTED

### 2.3. Patient Enrollment Criteria

The eligible patients were all confirmed as acute or chronic pulpitis or apical periodontitis by clinical and auxiliary examinations, with no previous dental pulp treatment, irregular diffuse radiography in the pulp cavity as shown by X-rays, and good openness. Besides, none used an analgesic medication in the previous 12 hours before taking part in the experiment. The age range was 18–60 years, and all patients had an educational level higher than middle school. Those with low treatment compliance, systemic diseases, or severe periodontitis were ruled out.

### 2.4. Methods

After the patients were admitted to hospital, they underwent cone beam computed tomography (CBCT) and routine full-mouth examination to determine the location, number, root canal orientation, and curvature of the affected teeth. The location and thickness of calcifications were determined by CBCT in CG, and the root canal was explored with # 10, # 8, and # 6 C-pilot files in turn. When the probe reached the deep part of the root canal or was stuck, the probe was rotated from side to side to continue to dredge down. Then, the G drill or a C-pilot file one size larger was utilized to manually dredge down until it was replaced with a # 15 C-pilot file for conventional root canal treatment. In RG, the root canal orifice was first probed with the DG16 probe, and then, the ET20 or ET40 working tip of the ultrasonic working instrument was used to remove the calcified tissue under the direct view of the microscope, with a depth of about 1-2 mm. After that, the root canal was gradually dredged with a C-pilot file or a # 8 manual K-file combined with a small amount of EDTA gel. If the calcified part was located in the lower segment of the root canal or the whole root canal was calcified, Hero642 or G drill would be used to open the middle and upper part of the root canal, followed by the use of the ultrasonic tip to remove the calcified tissue in this part. If the root canal was relatively straight, the ultrasonic working tip would be used to continue to dredge the root canal downward under the direct view of the DOM; for curved root canals, EDTA and C-pilot files would be used to repeatedly expand the root canal until the root canal was dredged. During the dredging process, the surface of the mouth mirror was wiped intermittently with 75% ethanol gauze or cotton balls. After the root canal dredging was completed, NiTi rotary file ProTaper was used to prepare root canal and the warm gutta-percha vertical condensation technique was utilized to complete root canal filling in both groups.

RETRACTED

### 2.5. Clinical Efficacy Evaluation

The clinical efficacy was assessed 6 months after treatment. Marked response: the symptoms disappeared, and the teeth could occlude normally, with no other abnormalities of the teeth as indicated by X-ray examination, no transmission area around the root apex of the affected tooth, and normal periodontal ligament space. Response: the symptoms were improved, and the teeth could occlude normally, but still with slight pain when chewing hard objects or hot and sour foods, and periodontal sparseness shown by X-rays. Nonresponse: the symptoms showed no improvement, with consciously irregular pain in patient, obvious masticatory disorder, sparse periodontal area by tooth X-rays, and projection area around the root apex. Overall response rate (ORR) = (marked response + response) cases/total number of cases × 100%.

### 2.6. Outcome Measures

(1) Dredging effect: it was assessed from dredging success rates of different tooth positions and calcification sites and total success rate. (2) Clinical efficacy. (3) Root canal dredging time. (4) Pain: it was evaluated by the Pain Intensity Numerical Rating Scale (PI-NRS) before (*T*0), during (*T*1), and after treatment (*T*2), and a higher score was associated with higher pain severity. The PI-NRS score includes mild pain (1–3), moderate pain (4–6), and severe pain (7–10). (5) Adverse reactions (ARs): the incidence of ARs including toothache, inability to eat, nausea and vomiting, and fever occurred within 1 week after treatment was calculated

### 2.7. Statistics and Methods

SPSS 22.0 statistical method was used to process the data. Count data were expressed as (percentages), and the intergroup differences were identified by the Chi-square test; the measuring data, denoted by mean ± standard deviation, were analyzed by the *t*-test (between-group) and ANOVA and LSD post hoc test (multigroup), with significance indicated by *P* < 0.05.

## 3. Results

### 3.1. Comparison of Patient Data

To ensure the accuracy of the experiment, general data such as age, BMI, gender, smoking, drinking, regular eating habits, long stay up late, tooth position, calcification site, and ethnicity were collected before the experiment for statistical analysis. It revealed no evident difference between groups (*P* > 0.05, Table 1), suggesting that the experimental results of the two groups of patients were comparable.

### 3.2. Comparison of Dredging Effect of Root Canal Calcification in Different Tooth Positions

The dredging success rates of anterior teeth, premolars, and molars and the overall dredging success rates of RG were 93.75%, 89.47%, 88.16%, and 89.23%, respectively, while those in CG were 61.54%, 71.43%, 73.91%, and 71.77%, respectively. The intergroup comparison revealed higher dredging success rates of root canal calcification in different tooth positions and a higher overall dredging success rate in RG compared with CG (*P* < 0.05, Table 2).

RETRACTED

### 3.3. Comparison of Success Rate of Root Canal Dredging in Different Calcified Sites

Then, comparing the root canal dredging of different calcified sites between the two groups, it can be seen that the success rate was also higher in RG than in CG (*P* < 0.05, Table 3). Among them, the overall dredging success rate of RG was 87.69%, with the dredging success rates of the upper root canal, the middle root canal, and the root apex being 91.30%, 78.95%, and 91.30%, respectively.

### 3.4. Comparison of Therapeutic Effects

Five patients in RG had ineffective treatment, and the ORR was 92.19%. In CG, 14 patients were ineffective, and the ORR was 79.41%. The intergroup comparison revealed a higher ORR in RG compared with CG (*P* < 0.05, Table 4).

### 3.5. Comparison of Dredging Time

The average dredging time of RG was 39.00 ± 7.36 min, which was statistically shorter compared with CG (51.90 ± 8.31 min) (*P* < 0.05, Figure 1).

### 3.6. Comparison of PI-NRS Scores

The two cohorts had similar PI-NRS scores at *T*0 (*P* > 0.05). Increased PI-NRS scores were found in both groups at *T*1, and the score in RG (4.36 ± 0.65) was significantly lower compared with that in CG (*P* < 0.05). At *T*2, both groups showed a lower PI-NRS score than *T*1 but higher than *T*0, and the score at *T*2 was also lower in RG (1.75 ± 0.69) as compared to CG (*P* < 0.05, Figure 2).

### 3.7. Comparison of Incidence of ARs

After treatment, 3 cases of toothache, 3 cases of inability to eat, and 2 cases of nausea and vomiting occurred in RG, with an overall AR rate of 12.50%. In CG, toothache, inability to eat, nausea and vomiting, and fever occurred in 7, 5, 4, and 2 cases, respectively, and the total AR rate was 26.47%. The intergroup comparison determined a lower incidence of ARs in RG (*P* < 0.05, Table 5).

## 4. Discussion

Root canal calcification is a defensive change of dental pulp tissue as the tooth ages and is stimulated by abrasion, inflammation, caries, etc. [9]. The formation of new protective tissues in the pulp cavity and inner wall of the root canal will also lead to root canal wall thickening and root canal obstruction [10]. Evidence has shown that the root canal calcification degree is generally related to different stimuli, and the closer the root canal is to the cavity, the more likely it is to calcify [11]. In addition, with the increase of age, dental pulp ages, restorative dentin and secondary dentine deposit, and the space of dental pulp cavity decreases, gradually increasing the number and degree of root canal calcification [12]. However, the operation of root canal dredging is difficult due to the special physiological structure of the mouth as well as the influence of operating instruments and surgical field of view, accompanied by large equipment consumption during the procedure and long operative time, which not only leads to strong discomfort in patients but also to high treatment cost that brings a greater economic pressure to patients [13]. This also makes root canal dredging a difficulty in the treatment of pulpal and periapical diseases. In clinical practice, it is urgent to find a safer, effective, and convenient treatment method to provide better medical services for patients.

RETRACTED

In this study, we compared the effects of traditional C-pilot files and mUS plus EDTA combined with C-pilot files in the treatment of root canal calcification. As it turned out, RG had better clinical curative effects and higher dredging success rates of different teeth positions and calcified parts than CG, suggesting excellent effects of mUS plus EDTA combined with C-pilot files in the treatment of root canal calcification. Moreover, we observed less dredging time and more significantly alleviated pain in RG, which once again demonstrated the important application potential of mUS plus EDTA combined with C-pilot files in root canal calcification.

In traditional root canal dredging, a small stainless steel C-pilot file is preferred for exploration, and then, the working tip of a C-pilot file with one size larger is utilized to manually dredge the root canal downward [14]. The use of the Pioneer file requires tentative dredging under the guidance of X-ray films and CBCT examination image data. Too insufficient a force can hardly achieve the dredging effect, while too strong a force may damage the pulp nerve of the patient, resulting in strong pain sensation [15]. Moreover, the working tip of the pilot file is easy to break into the dental pulp, which will not only affect the success rate of dredging but also require secondary treatment to take out the broken tip, further increasing the burden of patients [16]. Hence, the treatment of root canal calcification at the present stage has great limitations, which requires high operating experience, manipulation, and hand feeling of dentists. We speculate that this may be also the main reason for the lower success rate, longer time consumption, and obvious pain of patients in CG.

As an excellent imaging tool, CBCT can clearly display root canal curvature, calcification position, and degree, providing an accurate basis for clinical root canal treatment and effectively reducing the rate of root canal omission [17]. It is pointed out that with the assistance of CBCT, even an inexperienced stomatologist can achieve an ideal root canal preparation effect [18], which fully demonstrates the application value of CBCT for root canal calcification. However, with the development of minimally invasive medical technology, various minimally invasive microscopic instruments have been widely used in clinical practice. In recent years, it has been found that in the treatment of root canal calcification, the root canal microscope has a certain dual role of magnification and illumination, which can effectively improve the visual field clarity before operation, and plays an important role in promoting the root canal orifice, making up for the deficiency of traditional C-pilot files in tentatively searching for root canal orifice [19]. Furthermore, the root canal microscope can distinguish normal dentin from calcified root canals through subtle changes such as the color change of the dentin, effectively shortening the root canal evaluation time [20]. Therefore, combining ultrasonic instruments with root canal microscope can lead to effective identification of the location and degree of calcified lesions, allowing for quick removal of the calcified deposits on the root canal orifice and root canal by the cutting function and oscillation effect of ultrasonic instruments, thus improving the routine root canal exploration rate and the success rate of calcification removal. In this research, the root canal dredging effect of patients in RG was improved, which could verify this view. Besides, the reduction of ARs in RG corroborated the excellent safety of mUS plus EDTA combined with C-pilot files, which was of great significance for improving the treatment experience of patients.

RETRACTED

However, due to the short experimental cycle and the limited number of cases included, the prognosis of patients cannot be evaluated, which needs to be improved in future research. Besides, the therapeutic effect of root canal calcification may also have a certain potential relationship with the professional skills of dentists, so it is necessary to carry out root canal therapy training for dentists in our hospital to provide a more reliable guarantee for the treatment of patients.

## 5. Conclusion

EDTA combined with C-pilot files and mUS can effectively improve the dredging success rate of root canals obstructed by calcification, shorten the dredging time, improve patient comfort, and reduce the incidence of adverse responses, which is an effective method for clinical dredging of calcification obstructed root canals.

## Figures and Tables

**Figure 1:** Comparison of average dredging time. ^#^*P* < 0.05.

**Figure 2:** Comparison of PI-NRS scores. ^∗^*P* < 0.05 compared with the control group, ^#^*P* < 0.05 compared with *T*0, and ^&^*P* < 0.05 compared with *T*1.

**Table 1:** Comparison of patient data.

	Control group	Research group	*χ* ^2^ or *t*/*P*
Age	47.28 ± 4.53	46.34 ± 4.62	1.118/0.240
BMI (kg/m^2^)	27.05 ± 2.46	26.98 ± 2.67	0.157/0.876
Gender			0.008/0.931
Male/female	42/26	40/24	
Smoking			0.194/0.659
Yes/no	45/23	40/24	
Drinking			0.768/0.381
Yes/no	32/36	35/29	
Regular eating habits			0.089/0.765
Yes/no	28/40	28/36	
Long stay up late			0.040/0.841
Yes/no	32/36	29/35	
Tooth position (total calcified root canals 124/130)			0.707/0.702
Front teeth/premolars/molars	13/42/69	16/38/76	
o			0.922/0.631
Upper root canal/middle root canal/apex	62/43/19	69/38/23	
Nationality			2.889/0.089
Han/minority	65/3	64/0	

**Table 2:** Comparison of dredging effect of root canal calcification in different tooth positions.

	Anterior teeth	Premolars	Molars	Overall success rate
Control group	61.54 (8/13)	71.43 (30/42)	73.91 (51/69)	71.77%
Research group	93.75 (15/16)	89.47 (34/38)	88.16 (67/76)	89.23%
*χ* ^2^	4.535	4.060	4.843	12.420
*P*	0.033	0.044	0.028	<0.001

**Table 3:** Comparison of success rate of root canal dredging in different calcified sites.

	Upper root canal	Middle root canal	Root apex	Overall success rate
Control group	79.03 (49/62)	53.49 (23/43)	63.16 (12/19)	67.74%
Research group	91.30 (63/69)	78.95 (30/38)	91.30 (21/23)	87.69%
*χ* ^2^	3.966	5.781	4.896	14.700
*P*	0.046	0.016	0.027	<0.001

**Table 4:** Comparison of therapeutic effects.

	Marked response	Response	Nonresponse	Overall response rate (%)
Control group	24 (35.29)	30 (44.12)	14 (20.59)	79.41%
Research group	34 (53.13)	25 (39.06)	5 (7.81)	92.19%
*χ* ^2^				4.367
*P*				0.037

**Table 5:** Comparison of incidence of ARs.

	Toothache	Inability to eat	Nausea and vomiting	Fever occurred	ARs
Control group	7 (10.29)	5 (7.35)	4 (4.41)	2 (2.94)	26.47%
Research group	3 (4.69)	3 (4.69)	2 (3.13)	0 (0.0)	12.50%
*χ* ^2^					4.068
*P*					0.044

## Data Availability

The datasets used or analyzed during the current study are available from the corresponding author on reasonable request.
